The article "A Prognosis Marker Dynein Cytoplasmic 1 Heavy Chain 1 Correlates with EMT and Immune Signature in Liver Hepatocellular Carcinoma by Bioinformatics and Experimental Analysis" was published in 2022. Journal: Dis Markers.

# A Prognosis Marker Dynein Cytoplasmic 1 Heavy Chain 1 Correlates with EMT and Immune Signature in Liver Hepatocellular Carcinoma by Bioinformatics and Experimental Analysis

**DOI:** 10.1155/2022/6304859

**Published:** 2022-05-11

**Authors:** Yanhong Wang, Jiyu Han, Haichao Zhou, Songtao Ai, Daqian Wan

**Affiliations:** ^1^Department of Orthopedics, Tongji Hospital, School of Medicine, Tongji University, Shanghai 200065, China; ^2^Key Laboratory of Spine and Spinal Cord Injury Repair and Regeneration, Ministry of Education, Shanghai 200065, China; ^3^Department of Radiology, Shanghai Ninth People's Hospital, Shanghai Jiao Tong University School of Medicine, Shanghai 200011, China

## Abstract

**Background:**

Liver hepatocellular carcinoma (LIHC) has had a continuous increase in incidence and mortality rates over the last 40 years. Dynein Cytoplasmic 1 Heavy Chain 1 (DYNC1H1) is a protein coding gene which encodes the cytoplasmic dynein heavy chain family. This is the first investigation into the expression of DYNC1H1 and its mechanisms of action in LIHC patients.

**Methods:**

Based on the DYNC1H1 expression data from the TCGA database, we performed the DYNC1H1 expression, clinicopathological data, gene enrichment, and immune infiltration analysis. TIMER and CIBERSORT were used to assess immune responses of DYNC1H1 in LIHC. GEPIA, K-M survival analysis, and immunohistochemical staining pictures from the THPA were used to validate the results. In order to evaluate the diagnostic value of DYNC1H1, GEO datasets were analyzed by using ROC analysis. And quantitative real-time polymerase chain reaction was also carried out to evaluate the expression of DYNC1H1.

**Results:**

DYNC1H1 expression levels were associated with T classification, pathologic stage, histologic grade, and serum AFP levels. DYNC1H1 is an independent factor for a poor prognosis in patients with LIHC. Further study showed that high expression of DYNC1H1 was enriched in epithelial–mesenchymal transition (EMT) and the TGF *β* signaling pathway by GSEA analysis enrichment, indicating that DYNC1H1 might play a key role in the progression of CRC through EMT and immune response, which also had been validated by the experimental assays.

**Conclusions:**

DYNC1H1 will provide a novel and important perspective for the mechanisms of LIHC by regulating EMT. This gene will be able to act as an efficacious tool for the early diagnosis and effective intervention of LIHC.

## 1. Introduction

LIHC is one of the few prevalent solid organ tumors in which a continuous increase in incidence and mortality rates has been observed over the last 40 years [1]. The 2020 Global Cancer Statistics showed that LIHC new cases were approximately 906,000 and the death cases were 830,000, of which more than 50% occurred in China. Hepatocellular carcinoma (HCC) represents the predominant histological subtype (75–85%) of primary liver cancer [2]. Currently, several risk factors have been indicated to contribute for developing LIHC, such as hepatitis B, hepatitis C, excessive consumption of alcohol, exposure, tobacco use, and aflatoxin [3–5]. At present, ultrasonography (US), computed tomography (CT), magnetic resonance imaging (MRI), and the serum alpha-fetoprotein (AFP) value are the most common noninvasive methods used to detect and diagnose LIHC, but all of them are not always sufficiently sensitive in early diagnosis [6]. Therefore, the identification of a more specific biomarker and potential target for treatment is critical for improving the prognosis of LIHC.

Dynein Cytoplasmic 1 Heavy Chain 1 (DYNC1H1) is a protein coding gene which encodes the cytoplasmic dynein heavy chain family. This family links engulfment and execution of apoptosis to prevent several pathologies including cancer, neurodegenerative diseases, and autoimmune disorders [7–9]. The DYNC1H1 plays a dominant role in the assembly of the mitotic spindle and the congression of the metaphase plate [10]. DYNC1H1 also controls microtubule binding [11]. Therefore, DYNC1H1 involved in microtubule dynamics and mitotic spindle orientation could be a possible factor in the pathophysiology and progression of tumors [12]. They are closely linked to tumor pathogenesis [13, 14].

Although DYNC1H1-associated immune responses have been identified among various types of cancer, comprising gastric and lung cancer, the role of DYNC1H1 in immune infiltration and prognosis is still underexplored [11, 15]. To address this challenge, we analyzed DYNC1H1 in LIHC through using RNA expression sequencing data from The Cancer Genome Atlas (TCGA, https://cancergenome.nih.gov/) database. We used R language software to compare the interrelationship between DYNC1H1 and some clinicopathological parameters. In order to better confirm the pathogenic effect of DYNC1H1 and understand the regulatory mechanisms, we constructed protein–protein interaction (PPI) networks, Gene Ontology (GO) analyses, and gene set enrichment analysis (GSEA) analyses. The correlation between DYNC1H1 and EMT pathway scores was analyzed. Using the Tumor Immunoassay Resource (TIMER) and CIBERSORT algorithm, we further investigated the interrelationship between DYNC1H1 and Tumor-Infiltrating Immune Cells (TIICs). The association of DYNC1H1 and prognosis was subsequently analyzed by using the Gene Expression Profiling Interactive Analysis (GEPIA), Kaplan–Meier (K-M) survival analysis, and the Human Protein Atlas (THPA). In order to assess the diagnostic value of DYNC1H1, a receiver operating characteristic (ROC) curve was established. Finally, we further validated DYNC1H1 using qPCR, which will help us further elucidate the potential pathogenesis of LIHC.

Despite certain previous studies involving the potential role of this gene in LIHC [16, 17], the association of TIICs and poor prognosis did not present an exhaustive analysis and lacked an in-depth discussion. The development and pathogenesis of LIHC is an extremely complex process consisting of multiple causative aspects and risk factors involved in the etiology. Our study has suggested that higher DYNC1H1 expression is strongly associated with T classification, pathologic stage, histologic grade, AFP, and overall survival (OS) event, generally indicating a poor prognosis. In addition, the correlation between DYNC1H1 and TIICs was explored. In this paper, the function of DYNC1H1 in LIHC was analyzed in detail to explore effective molecules for LIHC diagnosis and treatment.

## 2. Materials and Methods

### 2.1. Data Acquisition and Mining

The TCGA database was utilized to find the gene expression data (workflow type: HTSeq-TPM), immune system infiltrates, and corresponding clinical information [18]. In addition, for any missing, insufficient, or unclear data source, the sample will be excluded from the research. We used both RNA-sequence and clinical data, which was used for analysis and investigation. Both RNA-sequence and relevant clinical data were used to guide further studies. Among these 424 cases, 374 cases of LIHC tissue and corresponding 50 cases of normal healthy liver tissues were included in our research. For investigation of the underlying molecular mechanism of the DYNC1H1 expression, patients with LIHC were clustered into 2 groups, the high or low expression level group based on patients' expression level and the median value of the DYNC1H1 gene. Our research was performed in conformity with the publication guidelines offered by TCGA [19]. Moreover, in order to verify the expression and diagnostic value of DYNC1H1 in LIH, we collected 2 gene expression profiling datasets (GSE14520 and GSE63898) from the Gene Expression Omnibus (GEO) database [20–22] (Table 1).

### 2.2. Validation of DYNC1H1 Expression

We analyzed the TCGA dataset to validate and verify the potential prognostic role of DYNC1H1 genes in LIHC. To analyze difference in DYNC1H1 genes between LIHC samples and normal liver tissues, we utilized independent sample *t*-tests for nonpaired samples and paired *t*-test for paired samples. The results were generated with boxplots. And using the ggplot2 R package [23], boxplots were plotted.

### 2.3. Survival Analysis Based on DYNC1H1 Expression

In short, using the R packages survival and survminer to graph K-M survival curves, survival analysis was carried out. It was the K-M survival curves that were used to represent the OS and progression-free interval (PFI) distributions between the high and low DYNC1H1 groups. By the OS and PFI time derived from TCGA, the relations of the DYNC1H1 expression level with patients' survival outcome was computed. Following that, in order to further appraise the upshots of the K-M survival analysis, receiver operating characteristic (ROC) curves were generated by using the pROC package [24] in R language [24].

### 2.4. Construction of the Predicted PPI Network

Using the DESeq2 R package [25], the samples were split into 2 expression groups in LIHC: low DYNC1H1 group (0–50%) and high DYNC1H1 group (50–100%). STRING, a well-known online biological tool for the prediction of PPI, comprises direct (physical) and indirect (functional) associations [26]. With the help of the version 11.0 of the PPI database STRING, we identified the differentially expressed genes (DEGs) involved in the PPI with the threshold values of |log2 fold − change(*FC*)| > 2.0 and adjusted *p* value (*p*.adjust) < 0.05. In this PPI network, the required interaction score for determining a significant interplay was medium confidence (0.400) as cut-off criteria. Second, the PPI network was visualized with Cytoscape (version 3.8.2) [27].

### 2.5. GO Pathway Enrichment Analysis of DEGs

GO analysis comprises a biological process (BP), cellular component (CC), and molecular function (MF). The GO enrichment analysis of DEGs in samples of LIHC was performed by the clusterProfiler [28] R package. Afterwards, we used the org.Hs.eg.db (version 3.4.0) and GOplot R (version 1.0.2) packages for analysis and visualization of the results by generating cluster plots [29].

### 2.6. Gene Set Enrichment Analysis

For GSEA, we chose normalized RNA-seq datasets from the TCGA data portal [30]. Herein, gene set permutations were set to 1000 with default parameters. Hallmark pathway enrichment analyses were performed to determine the possible biological function of DYNC1H1 by using GSEA. Enrichment results with 2 conditions (*p*.adjust < 0.05 and *q*-value <0.25) were considered as statistically significant.

### 2.7. Immune Infiltrate Analysis

TIMER is a comprehensive and publicly available resource for systemic analysis of immune infiltrates across various types of tumor (https://cistrome.shinyapps.io/timer/) [31]. We investigated the interrelation between the DYNC1H1 expression and the tumor using TIMER. The TIMER correlation module was also used to evaluate and visualize the interrelation between the gene and the tumor-infiltrating immune cell profile in LIHC. TIMER employs a previously released deconvolution statistical method to investigate associations among infiltrating immune cells and DYNC1H1 genes. We assessed the correlation between the expression of DYNC1H1 and the abundance of immune infiltrates (CD4+ T cells, dendritic cells, B cells, CD4+ T cells, B cells, neutrophils, and macrophages) in LIHC by the gene modules. The pictures of the gene against tumor purity were drawn using TIMER [32]. After that, to assess the relative gene expression, we chose a deconvolution algorithm called CIBERSORT (http://cibersort.stanford.edu/) on the basis of gene expression [33]. By evaluating the association between immune cell infiltration and DYNC1H1 expression in LIHC to uncover correlations between TIICs, we assessed the immune response of 24 TIICs by using CIBERSORT. We chose standard annotation files to build gene expression datasets by setting the default signature matrix at one thousand permutations. To determine the confidence of the deconvolution method, CIBERSORT derived a *p* value through Markov chain Monte Carlo (MCMC) methods. The three hundred and seventy-four tumor samples were classified into two groups to assess the significant effects of the DYNC1H1 expression on the microenvironment of the immune system. To identify the species of lymphocytes influenced by DYNC1H1, the *p* value < 0.05 was set up.

### 2.8. Comprehensive Analysis

The online database GEPIA analyzes the RNA-sequencing expression data of 8587 normal and 9736 tumor samples of 33 malignant tumors from TCGA and GTEx by using a standard processing pipeline [34]. OS with the DYNC1H1 expression in LIHC was analyzed by using GEPIA. Furthermore, a boxplot was generated to calculate the differential DYNC1H1 expression by using the tumor or normal state as a variable. Kaplan–Meier analysis of survival curve was performed using K-M survival analysis (http://kmplot.com/analysis/) to analyze interaction relationships between the DYNC1H1 expression and survival information with LIHC [35]. DYNC1H1 was fed into the database to graph K-M survival plots. The hazard ratio (HR) and the log-rank *p* value were calculated. Values with *p* value < 0.05 (*p* < 0.05) were considered to be statistically significant.

### 2.9. Immunohistochemistry-Based Validation of Hub Genes in THPA

THPA, a public database which includes over 5 million immunohistochemically stained tissues and cell distribution information for 26,000 human proteins, was a program supported by a grant from Sweden. THPA can examine normal and LIHC tissues via antibody proteomics, which is often used for the validation of the hub target genes' expressions. Therefore, we used this pathology tool to evaluate expression levels of DYNC1H1 between liver tissues and LIHC tissues from THPA.

### 2.10. Cell Culture

The human normal liver cell lines (L02) and hepatocellular carcinoma cell lines (Hep3B, HepG2, SMMC7721, and MHCC97H) were obtained from the Chinese Academy of Sciences (Shanghai, China). All cells were cultured in Dulbecco's modified eagle's medium (DMEM) containing 10% fetal bovine serum (FBS). Then after, cells were maintained in a humidified incubator containing 37°C and 5% CO_2_.

### 2.11. Quantitative Reverse-Transcription Polymerase Chain Reaction

According to the manufacturer's instructions, the total amount of RNA was extracted from the cell lines using a TRIzol reagent (Invitrogen, Thermo Fisher Scientific, Inc.) and subjected to reverse transcription using the PrimeScript™ RT Reagent Kit (Takara, Shiga, Japan). Quantitative Reverse-Transcription Polymerase Chain Reaction (qRT-PCR) was analyzed and performed using the Applied Biosystems® 7500 Fast Real-Time PCR System (Thermo Fisher Scientific, Waltham, MA) and accompanying Applied Biosystems® 7500 Software (version 2.0.6) to measure the mRNA expression levels of DYNC1H1. The following primer sequences were used: DYNC1H1 forward primer: TTGGGCACTAGGAAATTGATGC; DYNC1H1 reverse primer: GCAGGGTTGATACGCCACA.

### 2.12. Statistical Analysis

All statistical analyses were conducted using R statistical software (R Core Team, version 3.6.3). The univariate and multivariate models of the Cox analysis were used to show the multivariate HR and 95% confidence intervals (95% CI). We then evaluated the DYNC1H1 expression and other clinical and pathological features affecting OS. The significance threshold was set as probability (*p*) value < 0.05. Logistic regression was used to evaluate the associations between the DYNC1H1 expression and clinical characteristics (T stage, pathologic stage, histologic grad, AFP, and OS event). A *p* value of less than 0.05 was considered to be statistically significant.

## 3. Results

### 3.1. Survival Outcomes and Variable Analysis

To confirm the expression levels of DYNC1H1 in various species of tumors, we firstly analyzed the RNA-seq data from TCGA datasets using the TIMER tools. Analysis result shows that the expression level of DYNC1H1 is upregulated in the majority of tumors involving BLCA, CESC, CHOL, COAD, ESCA, GBM, HNSC, HNSC-HPV, KICH, KIRC, KIRP, LIHC, LUAD, LUSC, PAAD, PCPG, PRAD, SKUM, STAD, THCA, and UCEC (Figure 1(a)). To further validate the expression level and prognosis role of DYNC1H1 in these tumors, we checked their expression; we again analyzed the RNA-seq datasets and characteristics of the patient from the TCGA database and discovered that DYNC1H1 was upregulated when compared to all LIHC tissues and normal liver tissues (Figure 1(b)). We acquired the same outcome in paired LIHC tissues (*N* = 50) compared with normal liver tissues (Figure 1(c)). Meanwhile, the high expression of DYNC1H1 exhibited poor survival and progression-free survival of patients with LIHC (Figures 1(d) and 1(e)). As displayed in Table 2, we performed the Cox analysis to assess the correlation between the DYNC1H1 expression and overall survival, as well as other multivariable characteristics in LIHC patients. Univariate regression analysis demonstrated that a number of factors, comprising the pathologic stage (HR = 2.504, *p* value < 0.001), T stage (HR = 2.598, *p* value < 0.001), M stage (HR = 4.077, *p* value = 0.017), and DYNC1H1 expression (HR = 1.709, *p* value < 0.001), are highly associated with overall survival. The multivariate analysis, shown with a forest diagram in Figure 1(f), uncovered that the DYNC1H1 expression (*p* value = 0.009) is an independent factor for a poor prognosis in patients with LIHC (Table 2). The distribution of DYNC1H1 expression, survival status of patients with LIHC, and expression profiles of DYNC1H1 are depicted in Figure 1(g). The DYNC1H1 level displayed a robust prognostic value because the ROC curve indicated that the AUC of the DYNC1H1 expression for predicting survival was 0.704 (Figure 1(h)).

### 3.2. Relationship between DYNC1H1 Expression and Clinicopathology

Our study appraised the association between DYNC1H1 and clinicopathological characteristics of LIHC patients. The TCGA database includes 424 LIHC tissues including gene expression data and clinical characteristics obtained from LIHC patients. LIHC with increased DYNC1H1 expression was distinctly associated with T stage (*p* value < 0.05, Figure 2(a)), pathologic stage (*p* value < 0.01, Figure 2(b)), histologic grade (*p* value < 0.01, Figure 2(c)), AFP (*p* value < 0.01, Figure 2(d)), and OS event (*p* value < 0.001, Figure 2(e)). Results from this study showed that LIHC patients with high DYNC1H1 levels were more likely to present with worse T stage, worse pathologic stage, worse histologic grade, worse AFP, and worse OS event compared to those with low DYNC1H1 patients.

### 3.3. PPI Network Construction

In the PPI network, a total of 353 DEGs were included via the STRING database. The aim of the construction of the PPI network was to further understand the interactions of DEGs correlated with LIHC risk, including 180 nodes and 313 edges (Figure 2(f)).

### 3.4. GO Enrichment Analyses

In order to elucidate the mechanism of DYNC1H1 in the progression of LIHC, we performed GO enrichment analysis based on single-gene differential expression with the threshold values of |log2 *FC*| > 1.5 and *p*.adjust value < 0.05. GO functional analyses revealed these DEGs to be involved in biological processes including detoxification of copper ion (GO:0010273), stress response to copper ion (GO:1990169), detoxification of inorganic compound (GO:0061687), and stress response to metal ion (GO:0097501). In the molecular functions, the DEGs were primarily enriched in the receptor ligand activity (GO:0048018), ligand-gated ion channel activity (GO:0015276), ligand-gated channel activity (GO:0022834), and substrate-specific channel activity (GO:0022838). The cellular components of the DEGs were significantly enriched in the intrinsic component of the synaptic membrane (GO:0099240), immunoglobulin complex (GO:0019814), postsynaptic membrane (GO:0045211), and synaptic membrane (GO:0097060) (Table 3 and Figures 2(g) and 2(h)). The biological function and molecular role of DYNC1H1 were receptor-ligand, membrane, and immunoglobulin complex.

### 3.5. GSEA of DYNC1H1 in LIHC

In order to elucidate the mechanism of DYNC1H1 in the progression of LIHC, we then preformed GSEA to analyze the enrichment of the Hallmark pathways in the high-expression group and the low-expression group. Based on the NES, *q*-value, and *p*.adjust, significantly enriched Hallmark pathways were selected. When using the Hallmark gene set as a reference gene set, DEGs tended to be enriched in the following Hallmark signaling pathways: Hallmark epithelial mesenchymal transition, Hallmark estrogen response early, and Hallmark UV response DN, as depicted in Table 4 and Figure 2(i).

### 3.6. Regulation of the Progression of LIHC through the EMT Pathway

We found that the hallmark of EMT was the top of the enriched gene signature when comparing the high-expression group and the low-expression group from TCGA LIHC samples (Figure 2(j)). We next examined whether overexpression of DYNC1H1 affects EMT markers including SNAIL, SLUG, MMP9, TWIST1, and TWIST2 (Figure 2(k)). These findings suggest that DYNC1H1 might promote LIHC progression by regulating the EMT pathway.

### 3.7. Relationship between DYNC1H1 Expression and Tumor-Infiltrating Immune Cells

The presence of tumor-infiltrating lymphocytes (TIL) has emerged as an independent predictor of cancer sentinel lymph node status and overall survival rate (Azimi et al. 2012). We therefore chose the TIMER web tool to analyze the relationship between DYNC1H1 and the immune infiltration's level in LIHC. The results are shown in Figure 3(a). The expression levels of DYNC1H1 were positively correlated with the levels of B cells (*p* value = 3.51 × 10^−14^), CD8+ T cell (*p* value = 4.82 × 10^−7^), CD4+ T cell (*p* value = 3.91 × 10^−25^), macrophage (*p* value = 1.30 × 10^−28^), neutrophil (*p* value = 2.96 × 10^−24^), and dendritic cell (*p* value = 3.88 × 10^−22^). The aforesaid results showed that DYNC1H1 played a meaningful and pivotal role in immune infiltration. Furthermore, we sought to figure out whether the tumor immune microenvironment was distinct in LIHC patients with low DYNC1H1 compared to those with high DYNC1H1. According to the DYNC1H1 expression, the 424 tumor samples were classified into two groups, with 212 samples in the high expression of the DYNC1H1 group and 212 samples in the low-expression group. In order to further explore the mechanisms of immune response and the proportion of 24 immune cell populations in downloaded samples, we used the computational deconvolution method as implemented in CIBERSORT. Using the CIBERSORT algorithm, the difference between high and low DYNC1H1 expression groups in 24 immune cells was analyzed (Figure 3(b)). Plasmacytoid dendritic cell (pDC), CD56bright NK cells, macrophages, immature dendritic cells (iDC), eosinophils, dendritic cells (DC), cytotoxic cells, activated dendritic cells (aDC), T helper cells, central memory T cell (Tcm), effector memory T cell (Tem), T follicular helper cells (TFH), helper T type 1 (Th1) cells, and helper T type 2 (Th2) cells were influenced by DYNC1H1 levels, with notable variation existing in the dendritic cell and T cell lines between the high and low DYNC1H1 groups. Th2 cells, TFH, T helper cells, aDC, macrophages, and CD56bright NK cells were increased compared to the group with the low DYNC1H1 expression (*p* value < 0.001). Meanwhile, pDC, DC, and cytotoxic cells were decreased in the group with a high DYNC1H1 expression (*p* value < 0.001). In addition, we further examined possible correlations between 24 types of immune cells (Figure 3(c)). Moderate to strong correlations existed between different subpopulations of TIICs as per the heat map.

### 3.8. Data Validation

We first analyzed the mRNA expression of DYNC1H1 by using the GEPIA database. The DYNC1H1 level was increased in the LIHC group when compared to the normal control (Figure 4(a)). A significant interrelation was revealed between the high DYNC1H1 level and the poor OS for LIHC (*p* value = 3 × 10^−4^, Figure 4(b)). We further verified this finding by performing K-M survival plots. K-M survival plots showed that the high DYNC1H1 expression group was markedly correlated with poor overall survival rates (*p* value = 0.0049, Figure 4(c)). In addition, representative immunohistochemistry (IHC) images indicated that DYNC1H1 has higher expression levels compared to nontumor tissues from the THPA (Figure 4(d)).

### 3.9. DYNC1H1 Possesses a Higher Specificity than AFP for LIHC Diagnosis

Eventually, in order to evaluate the diagnostic value of DYNC1H1, GSE14520 and GSE63898 datasets were analyzed by using ROC analysis. As we know, alpha-fetoprotein (AFP) is a kind of diagnostic tumor marker that is commonly associated with LIHC. In GSE14520, the expression level of DYNC1H1 was significantly higher than that of the nontumor tissue (Figure 5(a)), and its AUC of 0.866 was higher than the AUC value of 0.685 for AFP (Figure 5(b)). In GSE63898, the expression level of DYNC1H1 was significantly higher than that of the nontumor tissue (Figure 5(c)), and its AUC of 0.796 was higher than the AUC value of 0.566 for AFP (Figure 5(d)). In Figure 5(e), the expression of DYNC1H1 was further validated by qRT-PCR in multiple cell lines.

## 4. Discussion

LIHC is the 3rd leading reason of cancer death and one of the five most frequently diagnosed cancer types [36]. During the past 20 years, LIHC's prevalence had been increasing persistently [37]. Cancer progression and metastasis have been implicated in a range of steps, including cell survival and proliferation, cell adhesion and migration, cell adhesion, and cell metabolism [38]. A number of previous biomarker studies have provided information on LIHC. Microtubule-associated serine and threonine kinase 2 (MAST2) was initially identified as a microtubule-associated protein. Recently, MAST2 is found to be a biomarker of diagnosis and prognosis of LIHC. The high expression level of MAST2 was correlated with advanced clinical status, for example, histological type, histologic grade, T classification, N classification, survival status, and poor prognosis of patients [39].

We assessed DYNC1H1 as a prognostic biomarker for LIHC in our current research. We evaluated the prognostic value of DYNC1H1 in patients with LIHC by analyzing the RNA-seq data from the TCGA database. Through DYNC1H1 analysis, and its interrelation to multiple tumor characteristics and immune cell responses, high DYNC1H1 expression served as an independent prognostic factor for poor OS. Furthermore, high DYNC1H1 expression levels were remarkably associated with T classification, pathologic stage, histologic grade, and serum AFP levels. Collectively, these results indicated that the DYNC1H1 expression level might influence LIHC initiation, progression, and immune microenvironment.

Subsequently, GO pathway analyses were performed. GO functional analyses revealed DYNC1H1 to be involved in biological processes including detoxification of copper ion, stress response to copper ion, detoxification of inorganic compound, and stress response to metal ion. The detoxification of inorganic compound like selenium plays a major role in tumor cell survival [40]. In parallel, these findings also indicate a close relationship between metal ions and immunity to cancer. This finding was in agreement with prior studies. Metal ion-activated immunotherapy is considered as an effective and potential approach in tumor therapy [41]. In the molecular functions, the DYNC1H1 was primarily enriched in receptor ligand activity, ligand-gated ion channel activity, ligand-gated channel activity, and substrate-specific channel activity. The family of ligand-gated channels warrants further investigation in tumor therapy [42–44]. The cellular components of the DYNC1H1 were significantly enriched in the intrinsic component of the synaptic membrane, immunoglobulin complex, postsynaptic membrane, and synaptic membrane. The synaptic membrane is complexed with tubulin which is essential for tumor cell migration [45].

GSEA was used as a method for determining pathway enrichment and functional module enrichment in the DEGs. Based on GSEA enrichment, we found that DYNC1H1 was involved in the EMT pathway and was positively correlated with EMT markers. Thus, it demonstrated that DYNC1H1 drove the EMT phenotype and regulated the EMT program in LIHC. This agreed with reality and was consistent with the importance of the EMT in HCC invasion and metastasis [46]. Additionally, the Hallmark results showed an enrichment in estrogen response early. In the literature, it is also suggested that antiestrogens or reduced estrogen levels may be linked to liver cancer [47].

In the present study, by using the TIMER database, we studied the connection between the DYNC1H1expression and the immune cell infiltration level in LIHC. It was found that DYNC1H1 was positively related with B cells, CD8+ T cells, CD4+ T cells, macrophages, neutrophils, and dendritic cells. Using the CIBERSORT algorithm, we confirmed that the high DYNC1H1 expression was related with the upregulation of Th2 cells, TFH, T helper cells, aDC, macrophages, and CD56bright NK cells and the downregulation of pDC, DC, and cytotoxic cells. DC serves as one of the functionally specialized antigen-presenting cells to play essential roles in initiating specific T cell responses for innate antitumor immunity [48]. It also regulated humoral immune responses to inhibit tumor development [49]. Therefore, we hypothesized that the function of DC could be suppressed by the overexpression of DYNC1H1. Summing up, these studies demonstrate that DYNC1H1 plays a critical role in modulating the immune responses of LIHC. However, randomized controlled trials (RCTs); multicenter randomized, controlled clinical trials, and mechanism researches are required for a more accurate understanding of the correlation between DYNC1H1 and LIHC in vitro and in vivo [50–52].

Finally, our results are validated by GEO datasets, its ROC curve analysis, and qRT-PCR. They demonstrated that the expression level of DYNC1H1 was significantly higher than nontumor tissue and its AUC was higher than the AUC value of AFP which was the mainstream biomarker for LIHC in 2 datasets. Altogether, these results showed that DYNC1H1 was expected to be the positive predictive tumor marker for patients with LIHC.

There are still several drawbacks to our research. The first point concerns data sources which come from public databases. In the future, we need to collect as many serum samples as possible from patients with LIHC, in order to validate this biomarkers. This brings us to the second point. Because the usefulness of biomarkers is mechanism dependent, we require more experimental validation and mechanistic elucidation in cell lines and animal models.

## 5. Conclusion

To sum up, DYNC1H1 associated with LIHC was identified using bioinformatic analysis. DYNC1H1 is a novel prognostic biomarker and has correlation with EMT and immune infiltrates in LIHC. With further study in the future, DYNC1H1 will provide novel and important perspectives for the mechanisms of LIHC. This gene will be able to act as an efficacious tool for the early diagnosis and effective intervention of LIHC.

## Figures and Tables

**Figure 1:** DYNC1H1 serves an oncogenic role in LIHC, and high DYNC1H1 expression predicts poor prognosis. (a) Human DYNC1H1 expression levels in different tumor types from TCGA database were determined by TIMER database (^∗^*p* < 0.05, ^∗∗^*p* < 0.01, and ^∗∗∗^*p* < 0.001). (b) The expression of DYNC1H1 in all LIHC samples from TCGA. (c) The expression of DYNC1H1 in paired CRC samples from TCGA. (d, e) The correlation between DYNC1H1 expression and survival status in TCGA. (f) Multivariate Cox analysis of DYNC1H1 expression and other clinicopathological variables. (g) DYNC1H1 expression distribution and survival status. (h) ROC curves of DYNC1H1.

**Figure 2:** DYNC1H1 expression was associated with clinicopathological features of LIHC based on TCGA and GO term/GSEA pathway enrichment results. Expression of DYNC1H1 correlated significantly with T stage (a), pathologic stage (b), histologic grade (c), AFP (d), and OS event (e). (f) PPI network. (g) *Z*-score results for the top 12 GO terms, including the top 4 BPs, CCs, and MFs. (h) Enrichment results for DEGs and the top 12 GO terms. (i, j) Gene set enrichment analysis. (k) The correlations between individual gene and EMT marker score.

**Figure 3:** Correlations between DYNC1H1 expression and immune infiltration levels in LIHC by TIMER. (a) Correlations between DYNC1H1 expression and immune infiltration levels. (b) The varied proportions of 24 subtypes of immune cells in high and low DYNC1H1 expression groups in tumor samples. (c) Heat map of 24 immune infiltration cells in tumor samples.

**Figure 4:** The synthesized analysis of DYNC1H1 mRNA expression and prognosis in patients with LIHC. (a) DYNC1H1 mRNA expression levels in normal and LIHC tissues, as obtained from GEPIA. (b) Levels of DYNC1H1 mRNA expression and overall survival based on data obtained from GEPIA. (c) Further validation of the correlation between DYNC1H1 expression and overall survival, as shown in K-M survival plot. (d) Hepatic expression of DYNC1H1 protein was visualized using immunohistochemistry via THPA.

**Figure 5:** DYNC1H1 shows a higher positive predictive value than AFP in LIHC patients. (a) The violin plot shows DYNC1H1 mRNA levels in patients with nontumor (*n* = 220) and LIHC (*n* = 225) from the GSE14520 dataset. (b) ROC curve analysis shows the diagnostic value of DYNC1H1and AFP in nontumor and LIHC patients from the GSE14520 dataset. (c) The violin plot shows DYNC1H1 mRNA levels in patients with nontumor (*n* = 168) and LIHC (*n* = 228) from the GSE63898 dataset. (d) ROC curve analysis shows the diagnostic value of DYNC1H1 and AFP in nontumor and HCC patients from the GSE63898 dataset. (e) DYNC1H1 expression level in LIHC by using qRT-PCR.

**Table 1:** Basic information of the microarray datasets.

ID	Platform	Data type	Author	Update date	Country	Sample type	*n* (*N*)	*n* (LIHC)
GSE14520	GPL3921	mRNA	Xin Wei Wang et al.	Oct 06, 2021	USA	Human tissues	220	225
GSE63898	GPL13667	mRNA	Augusto Villanueva et al.	Apr 14, 2020	USA	Human tissues	168	228

**Table 2:** Correlation between overall survival and multivariable characteristics in TCGA patients via Cox regression and multivariate survival model.

Characteristics	Total (*N*)	Univariate analysis		Multivariate analysis	
		Hazard ratio (95% CI)	*p* value	Hazard ratio (95% CI)	*p* value
Age	373				
≤60	177	Reference			
>60	196	1.205 (0.850-1.708)	0.295	1.314 (0.809-2.132)	0.270
Gender	373				
Female	121	Reference			
Male	252	0.793 (0.557-1.130)	0.200	1.062 (0.637-1.773)	0.817
Histologic grade	368				
G1 & G2	233	Reference			
G3 & G4	135	1.091 (0.761-1.564)	0.636	1.140 (0.709-1.834)	0.589
Pathologic stage	349				
Stage I & stage II	259	Reference			
Stage III & stage IV	90	2.504 (1.727-3.631)	<0.001	0.279 (0.015-5.202)	0.392
T stage	370				
T1 & T2	277	Reference			
T3 & T4	93	2.598 (1.826-3.697)	<0.001	9.921 (0.554-177.718)	0.119
M stage	272				
M0	268	Reference			
M1	4	4.077 (1.281-12.973)	0.017	2.200 (0.633-7.651)	0.215
N stage	258				
N0	254	Reference			
N1	4	2.029 (0.497-8.281)	0.324	3.437 (0.450-26.229)	0.234
DYNC1H1	373	1.709 (1.346-2.169)	<0.001	1.610 (1.128-2.297)	0.009

**Table 3:** Functional and pathway enrichment analyses for genes.

Ontology	ID	Description	Gene ratio	Bg ratio	*p* value	*p*.adjust	*q*-value
BP	GO:0010273	Detoxification of copper ion	10/555	15/18670	1.31*e*-12	2.41*e*-09	2.20*e*-09
BP	GO:1990169	Stress response to copper ion	10/555	15/18670	1.31*e*-12	2.41*e*-09	2.20*e*-09
BP	GO:0061687	Detoxification of inorganic compound	10/555	17/18670	8.02*e*-12	7.40*e*-09	6.74*e*-09
BP	GO:0097501	Stress response to metal ion	10/555	17/18670	8.02*e*-12	7.40*e*-09	6.74*e*-09
MF	GO:0048018	Receptor ligand activity	36/527	482/17697	4.32*e*-07	1.21*e*-04	1.04*e*-04
MF	GO:0015276	Ligand-gated ion channel activity	17/527	138/17697	7.58*e*-07	1.21*e*-04	1.04*e*-04
MF	GO:0022834	Ligand-gated channel activity	17/527	138/17697	7.58*e*-07	1.21*e*-04	1.04*e*-04
MF	GO:0022838	Substrate-specific channel activity	33/527	428/17697	6.50*e*-07	1.21*e*-04	1.04*e*-04
CC	GO:0099240	Intrinsic component of synaptic membrane	18/583	164/19717	1.83*e*-06	1.42*e*-04	1.23*e*-04
CC	GO:0019814	Immunoglobulin complex	20/583	159/19717	5.18*e*-08	1.95*e*-05	1.69*e*-05
CC	GO:0045211	Postsynaptic membrane	27/583	323/19717	1.35*e*-06	1.42*e*-04	1.23*e*-04
CC	GO:0097060	Synaptic membrane	33/583	432/19717	7.14*e*-07	1.34*e*-04	1.16*e*-04

**Table 4:** Signaling pathways most significantly correlated with DYNC1H1 expression based on NES, *q*-value, and *p*.adjust.

Hallmark pathways	Enrichment score	NES	*p*.adjust	*q*-values
Hallmark_epithelial_mesenchymal_transition	0.526697402	2.419142251	0.014927601	0.008485163
Hallmark_estrogen_response_early	0.432011711	1.988225556	0.014927601	0.008485163
Hallmark_UV_response_DN	0.443524891	1.954904884	0.014927601	0.008485163
Hallmark_angiogenesis	0.569576131	1.917856809	0.014927601	0.008485163
Hallmark_TGF_beta_signaling	0.521478423	1.906591073	0.01937609	0.011013777
Hallmark_mitotic_spindle	0.407384283	1.874883995	0.014927601	0.008485163

## Data Availability

The gene expression profiling data supporting this study are from previously reported studies and datasets, which have been cited. The expression and survival data are derived from TCGA and GEO databases. TCGA and GEO belong to public databases. The patients involved in the database have obtained ethical approval. Users can download relevant data for free for research and publish relevant articles. The qRT-PCR data used to support the findings of this study have not been made available.
